# Optimization of Sustainable Land Use Management in Water Source Area Using Water Quality Dynamic Monitoring Model

This article has been retracted.

**DOI:** 10.1155/2021/3881092

**Published:** 2021-12-09

**Authors:** Zhouyi Jin, Dabing Ge

**Affiliations:** ^1^College of Resources and Environment, Hunan Agricultural University, Changsha 410128, Hunan, China; ^2^Zhejiang College of Construction, Hangzhou 311231, Zhejiang, China

## Abstract

Land use management is the primary source of resource planning, and the management part of the sustainable ecosystem of water and soil resources is an important evidence for the sustainable development of the economic and social system. This is guided by the concept of sustainable development, and on the basis of the accumulation of relevant research practices and outcomes at home and abroad, water and land based systems are a research object and study the status of water and soil resource utilization, the state of water and soil coupling, and the supply and demand status of water resources. A balance analysis was carried out, and the gray linear programming model was used to optimize the allocation of land resources using the water quality dynamic monitoring model, which achieved the best coupling of water and soil resources and the greatest benefit. In this paper, aiming at the two types of problems in comprehensive water quality evaluation, namely, aiming at indifference and spatiotemporal changes, this article explores a powerful calculation method based on variable identification models and compiles a GIS geostatistical model (it is a computer-based tool that can draw and analyze ground objects; event GIS technology integrates seamless visual effects between map and local analysis services and general data processing services) to perform spatial analysis and visual expression of the evaluation results, in-depth analysis of the connotation, and theory and optimal allocation model of land resources optimal allocation. On the basis of the conceptual framework of the best share of land sources, the theories that should follow in the best share of land sources are discussed, and the available models and their characteristics are analyzed and compared. Experimental results show that, in the data provided by the analysis of water supply and demand balance at the annual spring system site by constructing an energy monitoring model, the water supply conditions of different water sources are rough, but the data of this study shows that the water shortage rate has reached 25%. In addition, the article explains the setting variables for the optimal allocation of land resources in water sources and compares and analyzes the optimization and planning of land resources in water sources.

## 1. Introduction

The land information system is driven by land management decision-making services and collects, manages, and operates land-related data in a computer software and hardware environment that integrates computer software technology, database technology, and GIS technology. With the rapid development of computer information technology, the development of land information systems will inevitably be synchronized with the development of computer information technology to promote the scientific and modernization of land resources management. Related researches on the optimal allocation of land resources mainly include theoretical research on optimal allocation of land resources and research on land resource evaluation techniques. The theoretical research on the optimal allocation of land resources can be roughly divided into two basic development stages: before the middle of the twentieth century, compared with urban planning, land use planning was a constructive or blueprint planning [1]. Since the 1970s, problems such as rapid population growth, resource shortages, and environmental pollution have increased in the world. In order to achieve the harmonious and sustainable development of population, resources, and the environment, land use planning has shifted from constructive planning to land control as the main means [2]. Under the premise of considering technical policies, economic society, and land environment, it emphasizes the combination of land use indicators and uses zoning to realize the sustainable use of population, land, water sources, environment, ecology, and other multiobjectives. Since then, land use planning has become a decision-making behavior. The optimal allocation of land resources can be embodied and implemented as its core content.

The theoretical research on the optimal allocation of land resources is mainly embodied in two aspects: land suitability evaluation and sustainable land use planning models. Land suitability evaluation believes that land use planning includes four basic contents: the general environment of the planning process, the subject of the planning process, the planning unit, and the level of completion of the planning [3]. It is an indicator to measure the degree of land use, which indicates the proportion of the land that has been used to the total land area, the larger the ratio, the higher the land utilization rate. There are indicators such as agricultural land utilization rate, nonagricultural land utilization rate, reclamation index, and multiple crop index. The research of land resource evaluation technology methods mainly focuses on the evaluation of agricultural land, and the main research content is the evaluation of land suitability and land potential. This is because traditional land use planning is the optimal allocation of agricultural land resources. Giri S et al. [4] established the soil correction coefficient in the evaluation of land production potential, so that the evaluation results can better reflect the level of land productivity. Kamali A [5] and others systematically studied land suitability evaluation methods based on intelligent computing and proposed methods such as fuzzy comprehensive evaluation models and neural network models for land suitability evaluation. Luo Y et al. [6] used fuzzy mathematics to revise the agroecological zone method proposed by FAO and applied GIS technology to the agroecological zone method.

This study takes sustainable land use in water source areas as the research object, evaluates the current situation of water and soil resource utilization and ways to change the unreasonable use of water and soil resources, and uses model analysis and planning methods to determine the optimal allocation of land resources under the constraints of water resources [7]. The distribution system is the general term for how labor products are divided among the social entities and the ration system. There is distribution according to work, distribution according to capital, distribution according to needs, and distribution in which multiple distribution methods coexist. This paper is based on a variable error identification model and a GIS hydraulic power rating. The overall status of water quality is determined by the many variables changing the water quality indicators. In assessing water quality, the interaction effect of multiple indicators and the confusing boundary between indicators and parameters should be considered. Therefore, this paper uses this model to measure the perfect water quality of a reservoir. In the statistical process, in order to obtain the reason and results of the thought analysis, this paper calculates the weight of each index based on the primary component analysis method. At the same time, due to the life-span of water quality, it is difficult to see the evolutionary characteristics of water quality under potent hydrological conditions such as rain and flow in common forms, linear charts, and GIS. Geostatistics methods include efficient world and visual analysis. Therefore, this paper introduces a comprehensive energy quality assessment method for water quality based on a combination of variable variance identification model and GIS and uses several methods to ensure the best quality of the combination of variable variance identification model and GIS for evaluation. Finally, combining the actual location and the importance of research on the optimal share of land resources, the model of optimal share of land resources under the constraints established by springs has been established. Under the constraints of the water quality energy monitoring model, the field function is built and solved by computer, and the optimization results are analyzed and compared. This paper explores a powerful evaluation method based on a variable identification model and combines the geostatistical model of GIS to analyze the world and visualize the evaluation results and analyze the deep interpretation, analysis, and subdivision model of the best share of land sources. Based on the introduction of the concept of the best share of land sources, the theories that should follow in the best share of land sources are discussed, and the available models and their characteristics are analyzed and compared.

The innovation of this article is that the article makes full use of the geostatistical model of GIS to conduct spatial analysis and visual expression of the evaluation results to construct a model between water quality detection and land management; it is a dynamic evaluation method based on a variable fuzzy recognition model. It can ensure the high accuracy of the data and experiments of the article, and the presentation of the data is more intuitive. Through this research, we can provide more efficient countermeasures for future land resource management.

## 2. Related Work

Water quality monitoring is an important basic work in water quality management, which mainly provides technical support for comprehensive water quality evaluation, water environmental protection and management by monitoring pollutants in water bodies, and their pollution factors [8]. The water quality monitoring work in my country was initially only for the chemical composition monitoring of natural river water. Later, with the emergence of water pollution problems, it began to add special water quality monitoring units to monitor some water pollution projects. So far, water quality monitoring work has been developed. In the rapid development stage, the water quality monitoring projects are constantly being supplemented and improved, and the monitoring technology is becoming more and more modern and standardized.

Water quality evaluation is based on water quality monitoring data, using reasonable methods to describe the quality of water bodies in accordance with the evaluation standards, thereby providing support for water environmental protection and rational use of water resources [9]. At the beginning of the 20th century, due to deterioration of river water quality, human water security could not be guaranteed, and water quality assessment work also developed accordingly. Water quality evaluation research in my country began in the 1950s. The initial research objects were only some major rivers and lakes (reservoirs). After recent years of development, water quality evaluation work has achieved many research results. Evaluation methods can quantify the comprehensive state of water quality and improve the efficiency of water quality management. In recent years, water quality evaluation methods have continued to develop and innovate. In terms of evaluation indicators, the initial physical and chemical indicators have gradually increased biological indicators, through a more comprehensive and scientific index system. Because there are many different water quality elements in the water body, such as total nitrogen, total phosphorus, and dissolved oxygen, these elements influence and restrict each other, and they are always in dynamic changes. At the same time, there are ambiguities and uncertainties in the evaluation process. In order to rationally quantify the comprehensive state of water quality, a large number of mathematical methods have been successively applied to water quality evaluation. These methods have their own characteristics and have solved the problem of comprehensive water quality to a certain extent. Several widely used methods are introduced below.

The single-factor evaluation method firstly compares the monitored values and standard values of each water quality index, obtains a separate water quality category for each index, and finally selects the worst water quality category among all the indicators as the final water quality evaluation result [10]. This method has clear thinking and simple operation and is currently used more, but its disadvantage is that it is too conservative and cannot fully reflect the comprehensive situation of water pollution. The evaluation process using the pollution index evaluation method is to first obtain the pollution index of the indicator by comparing the monitoring value and standard value of each water quality index and then use a mathematical calculation method to integrate the pollution index to obtain the comprehensive pollution of the water body. Different from the single-factor evaluation method, the evaluation result of the pollution index rating method represents the comprehensive situation of water quality pollution, but the evaluation result cannot reflect the dynamic changes of water quality.

Gray system theory takes into account the uncertainty and randomness of water quality and calculates water quality grades by constructing whitening functions and gray clustering matrices. Liu et al. [11] established a gray theoretical model for comprehensive evaluation of water quality based on the gray correlation degree, applied the model to groundwater quality evaluation in Qiqihar City, and concluded that the model is accurate, scientific, and reliable. Zhou et al. [12] used the gray clustering decision-making method to evaluate the surface water in a city and demonstrated the objectiveness and rationality of the method. Artificial neural network is to complete the evaluation of water quality through adaptive and self-organizing training by simulating the behavior characteristics of neural network. In Jiang et al. [13], artificial network technology was applied to the comprehensive assessment of the water quality of the first stream of the Fen River in Shanxi, and the probability of the method was demonstrated. Fan C et al. [14] used a synthetic network to measure groundwater quality and compare it with other methods, which showed that this method has a relatively high degree of accuracy when dealing with nonlinear problems such as rating.

Due to many uncertain factors in the water sector itself, and because the member relationship of water quality tests under multiple index conditions is also uncertain, Professor Chen Shouhuang gave the recommendations of the relative membership and the work of the related group and their development on this foundation. Process and method of identifying this variable confusion model is presented in [15]. Fuzzy boundary refers to focusing on the integration and synergy of internal and external resources, replacing the rigid structure model with a flexible organizational structure model, and replacing the original relatively fixed organizational structure with a sustainable structure. Since the variable fuzzy recognition model uses the relative membership degree to describe the membership of objective things, it effectively handles the fuzzy boundary problem between the index and the standard, realizes the simulation of the linear and nonlinear relationship between the elements by changing the model parameters, and makes the evaluation result more stable, so it has been widely used in water quality evaluation. For example, Li M et al. [16] used a variable fuzzy recognition model to calculate during the sea water quality evaluation and verified the accuracy of the method; Munthali MG et al. [17] evaluated the eutrophication of the water body based on the fuzzy recognition theory. The situation also yielded more accurate results. Kerr JM introduced a special chapter that focuses on promoting investment that produces environmental results, rather than investing in protection actions with unknown effects. Research based on fine-grained SWAT and other simulation models can guide the type, quantity, and location of protection investments to increase its impact on the environment [18]. Kroeger M reviewed the experience gained through the process of interdisciplinary integration in the sustainable land use research project in northeastern Germany and explored how and to what extent scenario development methods support the cognitive and social integration of interdisciplinary research groups [19].

## 3. Water Quality Dynamic Monitoring Model

The comprehensive state of water quality is determined by multiple water quality indicators that change dynamically. The essence of the water quality evaluation process is to compare the actual data obtained from monitoring with the evaluation standard value. Due to the continuous variability of the monitoring value, this comparison process is made. Any monitoring value is continuously subordinate to all levels and has the characteristic of “this and the other,” so if it is simply classified as a certain level, it will be inaccurate and not fully effective. The core idea of the variable fuzzy recognition model is to think that things have continuity and have the “this and other” in the classification process. This is consistent with the issues that should be considered in the water quality evaluation process, so this article adopts variable in fuzzy recognition model which conducts dynamic evaluation of water quality. At the same time, due to the changing time and life of water quality, in order to allow the evaluation results to directly reflect the time and evolutionary characteristics of water quality under powerful hydrological conditions such as rain and water flow, this discusses power and change of water quality. Water quality assessment method is based on variable variable identification model and GIS. The water quality dynamic monitoring model is shown in Figure 1.

The design objective of the mobile water quality monitoring system is to combine embedded technology and wireless communication technology to realize remote motion control and remote water quality monitoring functions of the mobile monitoring platform. Users can control the movement track of the mobile monitoring platform and view real-time water quality monitoring data and evaluation results through the monitoring center or handheld terminal. The 3G wireless communication module realizes data exchange with the monitoring center, sending the water quality information, GPS coordinate information, and electronic compass direction information obtained by the mobile water quality monitoring platform back to the monitoring center and at the same time receiving the control information sent by the mobile center.

### 3.1. Evaluation of Variable Fuzzy Recognition Model

In the process of comprehensive evaluation of water quality, it is necessary to consider the mutual influence between various indicators and the fuzzy boundary between indicators and standards. The variable fuzzy recognition model proposed by Professor Bai X [20] uses relative membership to deal with the dynamic changes of indicators, continuous membership, and fuzzy boundaries and can achieve linear and nonlinear simulations between variables by changing model parameters. Therefore, this paper uses variable fuzzy identification model to quantify the comprehensive evaluation level of water quality. The steps are as follows [21].

Suppose there are *n* water quality samples to be evaluated, and each sample is described by *m* index characteristic values. A sample can be represented by an index eigenvalue matrix *A* of type *m* x *n*, namely,

(1) $$\begin{array}{c} A_{m\times n}={\left\{a_{ij}\right\}}_{m\times n}=\left[\begin{array}{cccc} a_{11} & a_{12} & \ldots & a_{1n}\\ a_{21} & a_{22} & \ldots & a_{2n}\\ \ldots & \ldots & \ldots & \ldots \\ a_{m1} & a_{m2} & \ldots & a_{mn} \end{array}\right]. \end{array}$$

Among them, *a*_*ij*_ is the eigenvalue of the index *i* of sample *j*, *i*=1,2,…, *n*, *j*=1,2,…, *m*.

Identify and evaluate *n* samples according to the index standard values of *m* indexes and *c* levels to form an *m* x *n* type index standard eigenvalue matrix *Y*, that is,

(2) $$\begin{array}{c} B_{m\times n}={\left\{b_{ij}\right\}}_{m\times n}=\left[\begin{array}{cccc} b_{11} & b_{12} & \ldots & b_{1n}\\ b_{21} & b_{22} & \ldots & b_{2n}\\ \ldots & \ldots & \ldots & \ldots \\ b_{m1} & b_{m2} & \ldots & b_{mn} \end{array}\right]. \end{array}$$

Among them, *b*_*ij*_ is the modern parameter of index *i* level *j*, *i*=1,2,…, *m*, *j*=1,2,…, *l*.

Standardize the water quality evaluation samples and standards using standardized formulas (3) and (4), respectively,

(3) $$\begin{array}{c} p_{ij}=\left\{\begin{array}{cc} 0, & a_{ij}>b_{il}\;\mathrm{or}\;a_{ij}\leq b_{il},\\ \frac{\left(a_{ij}-b_{il}\right)}{\left(b_{i1}-b_{il}\right)}, & b_{il}>a_{ij}>b_{i1}\;\mathrm{or}\;b_{i1}\leq a_{ij}\leq b_{il},\\ 1, & a_{ij}\leq b_{i1}\;\mathrm{or}\;a_{ij}\geq b_{i1}, \end{array}\right. \end{array}$$

(4) $$\begin{array}{c} q_{ij}=\left\{\begin{array}{cc} 0, & b_{il}=b_{ik},\\ \frac{\left(b_{il}-b_{ik}\right)}{\left(b_{i1}-b_{ik}\right)}, & b_{ik}>b_{ij}>b_{i1}\;\mathrm{or}\;b_{i1}\leq b_{ij}\leq b_{ik},\\ 1, & b_{ij}=b_{i1}. \end{array}\right. \end{array}$$

Among them, *p*_*ij*_ is relative degree degree of water quality samples *j* index to the evaluation level; *q*_*il*_ is the normalized result of the *l-*level standard characteristic value of the index *i*; *k* is random variable between 1 to *l*.

After normalization, the sample set *A*_*mxn*_ is evaluated. Both are transformed into relative membership degrees between 0 and l, and the evaluation standard set Ymc is transformed into a cluster center between 0 and 1, and the two can be compared for level identification.

### 3.2. Dynamic Monitoring Index Weight Assignment

There are problems with the traceability algorithms applicable to the mobile water quality monitoring platform, so it is necessary to improve on the original basis or find a new algorithm to introduce it into the traceability of the mobile water quality monitoring platform. The principle of the particle swarm differential evolution algorithm is that birds forage for food, which is very similar to the traceability algorithm. Consider introducing the PSO-DE algorithm as the traceability algorithm for the mobile water quality monitoring platform [22]. The various water quality indicators of the water body represent the water quality status of the water body from different aspects, and their influence and contribution degree are different [23]. When combining multiple indicators to identify and quantify the quality of the body of water, it is necessary to choose the appropriate method to determine its contribution rate, that is, the indicator weight, and the normalized weight of each indicator is *W*={*w*_*ij*_}={*w*_1_, *w*_2_,…, *w*_*m*_} and satisfies ∑_*i*_^*n*^*w*_*i*_=1.

### 3.3. Determination of Comprehensive Water Quality Level

In order to better express the difference or distance between the water quality sample and the standards at all levels, the generalized index weight distance *s*_*ij*_ can be used to express

(5) $$\begin{array}{c} s_{lj}^{k}=\sum_{i=1}^{m}{\left(w_{i}\left|p_{ij}-q_{il}\right|\right)}^{k}. \end{array}$$

Among them, *w*_*i*_ is the weight of index *i*; *k* is the model parameter, which can be 1 or 2, respectively, representing the Hamming distance and Euclidean distance; the rest of the symbols are the same as before.

After obtaining the generalized index weight distance between the water quality sample and the standard, the comprehensive relative membership degree *g*_*ij*_ of the water quality sample *j* belonging to the water quality standard level *l* can be solved.

(6) $$\begin{array}{c} g_{lj}=\left\{\begin{array}{cc} 0, & l>b_{j}\;\mathrm{or}\;l<a_{j},\\ \frac{1}{\sum_{h=a_{j}}^{b_{j}}{\left(\sum_{i=1}^{m}{\left(w_{ij}\left(p_{ij}-q_{il}\right)\right)}^{k}/\sum_{i=1}^{m}{\left(w_{ij}\left(p_{ij}-q_{ih}\right)\right)}^{k}\right)}^{a/k},} & a_{j}\leq l\leq b_{j},\\ 1, & l=a_{j}=b_{i}. \end{array}\right. \end{array}$$

Among them, *l* is the water quality standard level; *a*_*j*_*b*_*j*_ are the lower limit and upper limit of the water quality sample level *j*; *w*_*i*_ is the weight of the index *i* of the water quality sample *j*; *a* is the parameter of the optimization criterion, which can be 1 or 2, respectively, representing the least-one-square criterion and the least-square criterion. By transforming model parameters *a* and *k*, different relationships between indicators and standards can be simulated. Under normal circumstances, *a* and *k* can have the following four relationships:

(7) $$\begin{array}{c} \left\{\begin{array}{c} a=1,k=1,\\ a=1,k=2,\\ a=2,k=1,\\ a=2,k=2. \end{array}\right. \end{array}$$

After calculating the comprehensive relative membership degree *g*_*ij*_ of the water quality sample level, substituting it into the grade characteristic value formula (4), the comprehensive evaluation level of the water quality sample *j* can be obtained.

(8) $$\begin{array}{c} G=\sum_{l=1}^{L}g_{lj}l. \end{array}$$

Among them, *G* is the characteristic value of the water quality sample level, that is, the comprehensive water quality status level; the rest of the symbols are the same as before. Substitute the standardized water quality samples and standards and index weights into formulas (4) and (5) to obtain the comprehensive water quality grade characteristic value, transform the model parameters *a, k*, and finally use the average of the 4 models as the comprehensive water quality evaluation result.

## 4. Optimization of Land Resource Allocation Model

Land use right refers to the unit or individual in accordance with the law or agreement. The rights include possession, use, profit, and limited disposal of state-owned land or collective land. The optimal allocation model of land resources is an important means to achieve optimal allocation, and a reasonable model plays an important auxiliary role in the optimal allocation of land resources. In view of this, the research on land optimization model has also made great progress [24]. The land resource optimization model is shown in Figure 2.

The system dynamics model is based on system theory, using computer simulation technology as a means, and adopts a combination of qualitative and quantitative structure-function simulation methods, emphasizing the analysis of system structure and less dependence on data. It is for simulating nonlinear dynamic feedback systems. It has a strong ability, which is significantly different from the linear programming model and other models. For example, Bai X uses the system's power model to compare and predict the relationship between the supply of urban land and the amount of land reservation, the difference between the supply and demand of urban land, and the overall intensity of the city to obtain the relationship between the supply and demand of urban land construction under different land intensiveness. At the same time, in the long-term simulation process, it is difficult to grasp the realities of the model, so this model is suitable for short- and medium-term conditions [25].

GIS comprehensive optimization model refers to the combination of mathematical methods and GIS technology, so that land resources can be optimized not only in quantity, but also in spatial structure, so that land resources can be scientifically managed and decided. With the support of GIS technology, Choi S K discussed the optimal allocation of land use on a larger regional scale based on land use zoning planning, suitability evaluation, and the establishment of linear programming models and realized the problem of land use optimization and the quantity and spatial optimal allocation of land resources within the county area. At the same time, the application of this model is also conducive to decision-makers to apply information technology to achieve a reasonable allocation of land resources.

Comprehensively consider the abovementioned land resource optimal allocation model and its characteristics and existing problems. At the same time, in order to maximize the benefit of land resource optimal allocation under water constraints, this paper adopts a method that combines linear programming model and gray system theory, namely, gray linear programming model. The use of gray theory can solve the problem of incomplete consideration of optimization objectives and constraints in linear programming. Therefore, gray linear programming model is selected to realize the optimal allocation of land resources under water constraints.

### 4.1. Water Demand Forecast

The water demand forecast in this paper is based on the economic and social development plan, taking 2018 as the current year of water resources analysis and forecasting water demand from three aspects: life, industry, and agriculture. Under the premise of considering the promotion of water-saving technologies, the status quo of water source areas, and the water supply capacity of the water supply project to be built, appropriate theories and methods are adopted to make quantitative and qualitative analysis of the future social water demand (Figure 3). According to the current situation of the water source area, we divide the water source area into three aspects: life, industry, and agriculture, and we forecast the water demand.

Based on the abovementioned forecasts of the economic and social development indicators of the water source area and the water demand standards of life, industry, and agriculture, the total water demand in the planned target year of the water source area is determined.

### 4.2. Water Providing and Requirements Balance

In the analysis of supply and demand demand, the demand for water and water in the proposed year is combined. According to the proposal mentioned above the annual water demand and local water analysis, the supply of springs and the demand balance of springs in 2020 are reflected in Figure 4.

### 4.3. Optimal Allocation Model of Land Resources under Water Resources Constraints

According to the current situation of land use and the problems in the spring area, the decision of the best course of land sources has been decided. Based on the gray line programming method, the gray line programming model is established and the decision variables are set. By setting a purpose function and setting the equilibrium equations with springs as the main constraint conditions, the optimal distribution of ground resources under different constraint constraints is obtained. The optimization results are compared and analyzed with the status quo and planning of land use to demonstrate the feasibility of the scheme and its effectiveness in the decision-making of sustainable use of water and soil resources.

### 4.4. Decision Variable Setting

According to the “National Land Use Status Classification Regulations” and the classification standards in the compilation of the overall land use plan, the land use types are set; this article is based on the land use status of city, and 11 variables are set, as shown in Figure 5.

### 4.5. Analysis of Optimization Results

According to the parameters and constraints determined above, the gray linear programming program is used to calculate the optimization results under different water resource constraints, as shown in Figure 6. According to the fuzzy comprehensive evaluation method, *w*_1_ = 0.1029, *w*_2_ = 0.1022, and *w*_3_ = 0.1297 are calculated, respectively. Therefore, the plan is the optimal configuration plan for the final screening, as shown in Figure 7.

### 4.6. Conclusion Discussion

Compare the results of optimized allocation of land resources under the constraints of water resources with the status quo and compare them with the planned land type structure, as shown in Figure 8. The analysis results: the optimized cultivated land area has been reduced, and the area of garden and forest land has been greatly reduced. The increase is consistent with the evaluation of land suitability, ecological planning, and the industrial policy for the development of winter jujube in the water source area; the increase in urban construction land and transportation water utilization land is relatively large, and the rural residential areas and mining land have been greatly reduced through consolidation and reclamation. It is conducive to the economical and intensive use of construction land; due to development and construction, the area of unused land is reduced by 6,685.48 hectares, while the area of waters and beaches remains unchanged before and after optimization. It can be seen that the optimized land type structure is more in line with the principle of intensive use. The utilization structure is more reasonable.

The data in the above figure is mainly a data simulation comparison between the current plan and the optimized plan, which covers natural resource protection, traffic water, industrial land, urban residential land, urban land, etc. In these aspects, optimized purchases planning can greatly save land resources and improve land management and allocation.

The optimization of water and land resources allocation indicators are implemented in space to effectively adjust the land use structure. The spatial allocation of the optimal plan is the overall optimization result of the city's land types, which is allocated to each township according to the water resources conditions to form an optimized land use planning map. The specific method is to modify the attribute table of the land use status database to modify the attributes of the land use type map spots that need to be converted, so that the map spot attributes of the land use planning type space are consistent with the optimization results.

## 5. Conclusion

This paper quantitatively analyzes the current situation of water and soil resource utilization from two aspects: comprehensive superiority of water and soil and index of water and soil resource. Revealing the contradiction between water and soil coupling in water source areas, it points out that, through optimized configuration, the benefit space of resource utilization can be greatly improved. Based on scientific research on the optimal share of land sources and analyzing the balance of water supply and demand, the procedures that should be followed in optimal share of land under the restrictions of springs are a move forward, and then the gray linear programming is used to establish an optimal allocation model for optimal solution, and a comparative analysis is made. The result is that the result of land use optimization can be used as a basis for land use planning and adjustment of land use structure. GIS software was used to configure the optimization results in space, so that the optimization plan was specifically implemented on the spatial plots, which solved the problem that the previous optimization of land allocation only solved the total amount of each type of land, but the spatial realization was more difficult. This article considers the objective factor of water resource constraints when configuring indicators for each land use type and overcomes to some extent the shortcomings of decomposing indicators that rely on human subjective judgments in current land use planning. The establishment of this method enriches the content system of technical specifications for land planning, incorporates objective constraints such as water resources into the basis for index decomposition considerations, considers the use of aggregation of land and springs, and promotes sustainable development. As an important part of the system, the monitoring center of the water quality monitoring system mainly realizes the processing of the data returned by the mobile water quality monitoring platform and then returns the control signal to the mobile platform. Through a large number of current domestic and foreign research statuses of sudden water pollution and mobile water quality monitoring system, the research investigates the status quo and explains the problems existing in the current mobile water quality monitoring system in China. However, the method used in the article is not yet able to solve the problem of high cost of water quality detection system. For this reason, the next work will be to trace a more comprehensive method, such as the two-dimensional water area suitable for small mobile water quality monitoring platform, and will research traceability algorithms.

## Figures and Tables

**Figure 1:** Water quality dynamic monitoring model.

**Figure 2:** The basic idea of establishing a land resource optimization model.

**Figure 3:** Predicted results of the planned target annual water demand in the water source area.

**Figure 4:** Water supply and demand balance for planning target year in water source area.

**Figure 5:** Description of setting variables for optimal allocation of land resources in water source areas.

**Figure 6:** Alternative plan units for optimal partition of land resources in water source areas.

**Figure 7:** Best results of land sources under water resources restrictions in spring.

**Figure 8:** Comparative analysis of land resource optimization and planning in water source areas.

## Data Availability

The data used to support the findings of this study are available from the corresponding author upon request.

## References

[1] Geng R., Sharpley A. N. (2019). A novel spatial optimization model for achieve the trad-offs placement of best management practices for agricultural non-point source pollution control at multi-spatial scales. *Journal of Cleaner Production*.

[2] Xu H., Brown D. G., Moore M. R., Currie W. S. (2018). Optimizing spatial land management to balance water quality and economic returns in a Lake Erie watershed. *Ecological Economics*.

[3] Xie H., Zhang Y., Zeng X., He Y. (2020). Sustainable land use and management research: a scientometric review. *Landscape Ecology*.

[4] Giri S., Qiu Z., Zhang Z. (2018). Assessing the impacts of land use on downstream water quality using a hydrologically sensitive area concept. *Journal of Environmental Management*.

[5] Kamali A., Niksokhan M. H. (2017). Multi-objective optimization for sustainable groundwater management by developing of coupled quantity-quality simulation-optimization model. *Journal of Hydroinformatics*.

[6] Luo Y., Yang K., Yu Z. (2017). Dynamic monitoring and prediction of Dianchi Lake cyanobacteria outbreaks in the context of rapid urbanization. *Environmental Science and Pollution Research*.

[7] Gu Q., Hu H., Ma L. (2019). Characterizing the spatial variations of the relationship between land use and surface water quality using self-organizing map approach. *Ecological Indicators*.

[8] Dissanayake D., Morimoto T., Ranagalage M. (2019). Accessing the soil erosion rate based on RUSLE model for sustainable land use management: a case study of the Kotmale watershed, Sri Lanka. *Modeling Earth Systems and Environment*.

[9] Nguyen H. H., Recknagel F., Meyer W., Frizenschaf J., Shrestha M. K. (2017). Modelling the impacts of altered management practices, land use and climate changes on the water quality of the Millbrook catchment-reservoir system in South Australia. *Journal of Environmental Management*.

[10] Messina N. J., Couture R.-M., Norton S. A., Birkel S. D., Amirbahman A. (2020). Modeling response of water quality parameters to land-use and climate change in a temperate, mesotrophic lake. *The Science of the Total Environment*.

[11] Liu J., Shen Z., Chen L. (2018). Assessing how spatial variations of land use pattern affect water quality across a typical urbanized watershed in Beijing, China. *Landscape and Urban Planning*.

[12] Zhou X.-Y., Lei K., Meng W., Khu S.-T. (2017). Industrial structural upgrading and spatial optimization based on water environment carrying capacity. *Journal of Cleaner Production*.

[13] Jiang Y., Yang X., Liang P., Liu P., Huang X. (2018). Microbial fuel cell sensors for water quality early warning systems: fundamentals, signal resolution, optimization and future challenges. *Renewable and Sustainable Energy Reviews*.

[14] Fan C., Chen K.-H., Huang Y.-Z. (2021). Model-based carrying capacity investigation and its application to total maximum daily load (TMDL) establishment for river water quality management: a case study in Taiwan. *Journal of Cleaner Production*.

[15] Shrestha S., Bhatta B., Shrestha M., Shrestha P. K. (2018). Integrated assessment of the climate and landuse change impact on hydrology and water quality in the Songkhram River Basin, Thailand. *The Science of the Total Environment*.

[16] Li M., Fu Q., Singh V. P., Liu D., Li T. (2019). Stochastic multi-objective modeling for optimization of water-food-energy nexus of irrigated agriculture. *Advances in Water Resources*.

[17] Munthali M. G., Mustak S., Adeola A., Botai J., Singh S. K., Davis N. (2020). Modelling land use and land cover dynamics of Dedza district of Malawi using hybrid Cellular Automata and Markov model. *Remote Sensing Applications: Society and Environment*.

[18] Kerr J. M., Depinto J. V., Mcgrath D., Sowa S. P., Swinton S. M. (2016). Sustainable management of Great Lakes watersheds dominated by agricultural land use. *Journal of Great Lakes Research*.

[19] Kroeger M., Schaefer M. (2016). Scenario development as a tool for interdisciplinary integration processes in sustainable land use research. *Futures*.

[20] Bai X., Jia X., Jia Y., Shao M. a., Hu W. (2020). Modeling long-term soil water dynamics in response to land-use change in a semi-arid area. *Journal of Hydrology*.

[21] Choi S.-K., Jeong J., Kim M.-K. (2017). Simulating the effects of agricultural management on water quality dynamics in rice paddies for sustainable rice production-model development and validation. *Water*.

[22] Song M., Cui X., Wang S. (2019). Simulation of land green supply chain based on system dynamics and policy optimization. *International Journal of Production Economics*.

[23] Wu J.-H., Wei W., Zhang L. (2019). Risk assessment of hypertension in steel workers based on LVQ and Fisher-svm deep excavation. *IEEE Access*.

[24] Li C., Sun L., Xu Z., Wu X., Liang T., Shi W. (2020). Experimental investigation and error analysis of high precision FBG displacement sensor for structural health monitoring. *International Journal of Structural Stability and Dynamics*.

[25] Zhang K., Wang Q., Chao L. (2019). Ground observation-based analysis of soil moisture spatiotemporal variability across a humid to semi-humid transitional zone in China. *Journal of Hydrology*.

